RETRACTED

# Laparoscopic Radical Resection versus Routine Surgery for Colorectal Cancer

**DOI:** 10.1155/2022/4899555

**Published:** 2022-09-30

**Authors:** Yan Chen, Dong Xi, Qiutao Zhang

**Affiliations:** ^1^Department of General Surgery, Changzhou Wujin People's Hospital, Changzhou, Jiangsu, China; ^2^Wujin Clinical College, Xuzhou Medical University, Changzhou, Jiangsu, China

## Abstract

For patients with colorectal cancer, minimally invasive surgical methods, particularly laparoscopic methods, are now the preferred course of therapy. This research is performed to investigate the effects of laparoscopic radical resection on patients with colorectal cancer. A total of 100 colorectal cancer patients treated in our hospital from January 2017 to January 2019 were enrolled. The subjects were divided into observation (*n* = 50) and control (*n* = 50) groups and treated with laparoscopic surgery and laparotomy, respectively. As well as postoperative complications and survival rates, the levels of inflammatory substances, stress response, immunological function, and perioperative markers were compared between the two groups. There was no significant difference in the postoperative exhaust time between the two groups (*P* > 0.05). Compared with the control group, the observation group showed longer operation time, faster recovery of intestinal function, shorter hospital stay, and less intraoperative bleeding amount (*P* < 0.05). The serum contents of hs-CRP, TNF-*α*, IL-6, norepinephrine, adrenaline, and cortisol at 1 d, 3 d, and 5 d after surgery were significantly higher than before in both groups (*P* < 0.05). Moreover, the serum contents of hs-CRP, TNF-*α*, IL-6, norepinephrine, adrenaline, and cortisol in the observation group were significantly lower than that in the control group (*P* < 0.05). At 10 days following surgery, immune index levels had dramatically increased in both groups, with noticeably higher immune index levels in the observation group than in the control group (*P* < 0.05). There were no appreciable differences in the two groups' 2-year survival rates (*P* > 0.05), but the complication rate was much greater in the control group (*P* < 0.05). To sum up, after laparoscopic surgery, patients had fewer complications, shorter hospital stay, lower inflammatory factor expression, less stress response, better immune function, less trauma, faster recovery, and improved quality of life.

## 1. Introduction

Colorectal cancer is a common clinical gastrointestinal malignant tumor, including colon cancer and rectal cancer. With the improvement of people's living standards and the changes of diet structure in recent years, the incidence rate of colorectal cancer is increasing by year [1, 2]. Colorectal cancer patients are usually asymptomatic or almost asymptomatic in the early stage. As the condition progresses, symptoms such as altered bowel habits, hematochezia, abdominal pain, abdominal mass, intestinal blockage, and other symptoms may appear. The majority of these symptoms require surgical resection as a form of treatment [3, 4]. The use of minimally invasive surgical methods, particularly laparoscopic methods, has advanced significantly in clinical practice and is now the treatment of choice for people with colorectal cancer. Laparoscopic radical resection for colorectal cancer provides equivalent efficacy to standard laparotomy with the advantages of less trauma, quicker recovery, and higher safety [5, 6].

RETRACTED

The new procedure method of laparoscopic surgery is based on the old procedure method of laparoscopic surgery. Its primary feature is to minimize laparoscopic ports and eliminate dangers such problems from intravenous needles. Nevertheless, the operation's clinical application duration is brief. Whether it shares the same effect with traditional porous laparoscopic surgery or reduces the harm to patients is not fully clear [7, 8]. The purpose of the current study was to ascertain the safety of laparoscopic radical resection for colorectal cancer and how it affected patients' prognoses for survival.

## 2. Clinical Information and Methods

### 2.1. General Clinical Data

A total of 100 patients treated in our hospital from January 2017 to January 2019 were selected as research objects and divided into observation and control groups with 50 patients each. They were treated with laparoscopic surgery and laparotomy, respectively, according to principles from The Guidelines for Colorectal Cancer. Among the 50 cases in the observation group, 2 cases were found to be in the terminal stage and were closed with abdomen (1 extensive peritoneal metastasis and 1 mesenteric metastasis in the small intestine), and 1 case was converted to laparotomy (locally advanced carcinoma with invasion of the small intestine). Forty-seven cases were actually included in the study, including 25 men and 22 women, aged within 56.3 ± 11.5 (32~74 years old). Among the 50 patients in the control group, 2 patients had distant metastasis of cancer (1 patient had multiple small metastases in left and right liver and 1 patient had multiple peritoneal metastasis). Forty-eight patients were actually included in the study, including 22 men and 26 women, aged within 57.1 ± 8.1 (33~76 years old). The patients with TNM stages of 0 to 1, 2, and 3 in observation and control groups were 16, 17, and 14 and 17, 16, and 15, respectively. The differences of the age, sex, and disease stage between the two groups had no statistical significance (*P* > 0.05), which proved that the two groups are comparable. Inclusion criteria are as follows: (1) no distant organ metastasis diagnosed by CT and other preoperative imaging and (2) colorectal cancer by colonoscopy and pathological examination and were all deadline surgery. Exclusion criteria are as follows: (1) history of major abdominal surgery, (2) acute diseases such as concurrent intestinal obstruction and intestinal perforation, (3) history of malignant tumors in other parts, and (4) history of radiotherapy or chemotherapy before surgery. The study was approved by the ethics committee of Changzhou Wujin People's Hospital, with informed consent from either the patients or the family members.

RETRACTED

### 2.2. Treatment Methods

Patients in the control group routinely received open surgery. One day before surgery, the patients took antibiotics and compound polyethylene glycol electrolyte powder as intestinal preparation, fasted for solids 8 h before surgery, fasted for liquids 4 h before surgery, and emptied bladder before surgery. The patient was placed in the supine position or bladder lithotomy position with general anesthesia and endotracheal intubation. The 12 to 15 cm abdominal incision was made and separated by layer. According to the intraoperative exploration, the operation method is determined: D3 complete mesorectal excision for colon cancer and D3 total mesorectal excision for rectal cancer [4]; after colorectal cancer resection and digestive tract reconstruction, the abdominal cavity was washed and checked with no bleeding. The drainage tube was retained and the incision was closed.

The laparoscopic surgery procedure was offered to the observation group. The control group's preoperative planning and anaesthesia were used. Patients were lying on their backs with their legs parted or in a low lithotomy position. On the left lower abdomen, a 2-4 cm long incision was created [5]. Carbon dioxide pneumoperitoneum was established with pressure controlled at 12~14 mmHg (1 mmHg = 133.3 Pa). Laparoscopy was placed into the abdominal cavity using five-port method. The surgery type was determined according to the laparoscopic detection: D3 laparoscopic complete mesorectal excision for colon cancer and D3 laparoscopic total mesorectal excision for rectal cancer. After laparoscopic cancer free and lymph node dissection, a small incision (6-8 cm) was made in the abdomen to help complete the resection of the colorectal cancer lesions. The intestines with colon cancer except sigmoid colon were placed back into the abdominal cavity after the reconstruction of the digestive tract outside of the small incision. The pneumoperitoneum was rebuilt. No bleeding was found after cleaning and inspecting the abdominal cavity. The incision was closed after keeping the drainage tube. After a 6 to 8 cm long colorectal cancer lesion was removed in cases of sigmoid colon or rectal cancer, the pneumoperitoneum was reconstructed. The anastomosis was completed in the abdominal cavity with the aid of laparoscopy. All postoperative patients received the same care.

RETRACTED

### 2.3. Observation Indexes

1. Perioperative period, including operation time, intraoperative bleeding volume, borborygmus recovery time, postoperative exhaust time, and hospital stay
2. The occurrence of complications in 2 groups, including incision infection, anastomotic leakage, bleeding, and urinary infection
3. Inflammatory factors: before and 1 d, 3 d, and 5 d after the surgery, 8 mL of venous blood was collected and centrifuged at 3500 r/min for 10 min. The upper serum was stored in a freezer for detection of high-sensitive C reactive protein (hs-CRP), tumor necrosis factor-*α* (TNF-*α*), and interleukin-6 (IL-6) using R&D enzyme-linked immunosorbent assay (ELISA) kits. The ELISA kit was provided by Shanghai Yanjin Biotechnology Co., Ltd
4. Stress response: four mL of upper serum samples was retained and analyzed, including the content of norepinephrine (NE), epinephrine (E), and cortisol (Cor). The ELISA kit used was provided by Shanghai Yanjin Biotechnology Co., Ltd
5. IgG, IgM, and IgA levels were measured by ELISA. Detection reagents were produced and provided by Shanghai Enzyme-Linked Biotechnology Co., Ltd., CD4 and CD8 were measured using flow cytometer (model CytoFLEX), and the proportion of CD4/CD8 was calculated
6. Survival rate and recurrence rate: after 2 years of postoperative follow-up, the total postoperative survival rates of the two groups of patients were compared. The follow-up started after the surgery and ended in November 2020

### 2.4. Statistical Analysis

Statistical analysis was performed using SPSS 18.0 software. The measurement data was expressed as *x* ± *s* with *t*-test used for intergroup comparison. *X*-test was used for intergroup comparison of enumeration data. *P* < 0.05 indicates statistical significance.

## 3. Results

### 3.1. Comparison of the Perioperative Conditions between the Two Groups

There was no significant difference in postoperative exhaust time between the two groups (*P* > 0.05). Compared with the control group, the observation group showed longer operation time, shorter recovery time and hospital stay, and less intraoperative bleeding (*P* < 0.05), as is shown in Table 1.

### 3.2. Comparison of Serum Inflammatory Factor Levels before and after Surgery between the Two Groups

Both groups showed higher postoperative levels of hs-CRP, TNF-*α*, and IL-6 than preoperative (*P* < 0.05). Their levels were gradually reduced on the third and fifth days. The observation group has lower levels of hs-CRP, TNF-*α*, and IL-6 than the control group on the first, third, and fifth days (*P* < 0.05). The outcomes are shown in Figure 1.

RETRACTED

### 3.3. Comparison of Stress Responses before and after Surgery between the Two Groups

The postoperative levels of NE, E, and Cor were significantly higher than preoperative at 1 d, 3 d, and 5 d (*P* < 0.05). Compared with the control group, the observation group showed lower levels of NE, E, and Cor at 1 d, 3 d, and 5 d (*P* < 0.05). The results are shown in Figure 2.

### 3.4. Comparison of Immune Indexes before and 10 d after Surgery between the Two Groups

There were no significant differences in the preoperative immune indexes between the 2 groups (*P* > 0.05). The postoperative immune indexes were strangely increased in both groups and were higher in the observation group than the control group with statistical significance (*P* < 0.05). The results are shown in Figure 3.

### 3.5. Comparison of Complication Rates between the Two Groups

The results showed that the incidence rates of complications in the control group were significantly higher, with statistically significant differences, compared with the observation group (*P* < 0.05), as shown in Table 2.

### 3.6. Comparison of 2-Year Postoperative Survival between the Two Groups

There were no significant differences in the postoperative overall 2-year survival rates between the 2 groups (*P* > 0.05), as is shown in Figure 4.

## 4. Discussion

Colorectal cancer is a common clinical malignant tumor. One study in 2016 has shown that there are 159,000 deaths of colorectal cancer per year. Its morbidity and mortality rank the fifth among malignant tumors in China. The number of new patients per year ranks the 4th, about 331,000. The economic development, improvement of living standard, and transformation of diet structure are important factors leading to the incidence and death of colorectal cancer [9]. At present, surgery is the only successful treatment and cure for colorectal cancer. Before the widespread use of laparoscopic surgery, traditional laparoscopic surgery was the most commonly used surgery, which could completely remove lymph nodes and tumors [10, 11]. However, laparotomy also has disadvantages such as excessive bleeding, large trauma, high infection rate, and slow postoperative intestinal function recovery. Since laparoscopic colectomy was proposed by Jacobs et al. in 1991, it has gradually been popularized in the treatment of colorectal cancer and becomes the classic way of surgery [12]. The amplification effect of laparoscopic images can broaden the surgical field, facilitating the operator to identify the important structure of blood vessels, nerves, and ureter more clearly, thus to clean the lymph nodes more thoroughly and protect the nerves. This operation is more accurate, especially for obese patients or male patients with a relatively narrow pelvis requiring pelvic surgery, with considerable advantages over laparotomy [5, 13, 14].

RETRACTED

By examining perioperative indicators, we discovered in this study that traditional open surgery and laparoscopic surgery had similar therapeutic outcomes, including complete mesentery excision and a negative circumferential margin, which is similar to some prior findings [15]. Our research demonstrated that laparoscopic surgery patients experienced less intraoperative bleeding, a shorter hospital stay, and longer surgical times. The lengthy procedure time is a result of the laparoscopic colorectal surgery's complexity and extensive learning curve. One study [16] found that as operator experience accumulated, operative time for laparoscopic surgery tends to be shortened. Moreover, due to the small incision, the intraoperative bleeding volume is reduced and the postoperative recovery time is shortened.

A type of invasive surgery called laparoscopic surgery undoubtedly have an effect on the patient's body, which largely shows up as the production of numerous inflammatory cells and a heightened stress reaction, among other things [17, 18]. The hs-CRP is an important indicator reflecting the inflammatory state of the body, which can increase in several hours after the tissue damage and peak within 48 h. With the remission of the body damage, its expression gradually reduces [19]. TNF-*α* is regarded as the most potent marker of endogenous inflammation in the body because of its role as a monocyte cell factor in triggering and starting local inflammatory responses [20]. IL-6 is an early reaction substance of acute phase injury, which belongs to a class of proinflammatory factors, and its elevation degree is positively correlated with the inflammatory response [21]. NE, E, and Cor are representative stress factors released by the body under the stress response. Their facial expressions can quickly change in reaction to events like surgery, which is directly correlated with the intensity of the body's stress response. In this study, patients treated with laparoscopic surgery had lower hs-CRP, TNF-*α*, IL-6, NE, E, and Cor levels at 1 d, 3 d, and 5 d than those with conventional laparotomy, suggesting that laparoscopic surgery reduces tissue damage induced by multiple incisions and avoid drastic increase in postoperative inflammatory factors and stress indicators, compared with traditional laparotomy.

RETRACTED

T lymphocytes mediate cellular immune function. CD+3, CD+4, CD+8, and CD+4/CD+8 play important auxiliary roles in the immune process, which can reflect the immune regulation state of the body, which is related to [22, 23] the long-term prognosis of patients. The results of this study showed that compared with preoperative levels, the postoperative levels of IgA, IgG, IgM, and CD+4/CD+8 were strangely increased in both groups. The improvement in the observed group was significantly better than that in the control group. It demonstrated that physical trauma from surgery lowers the intensity of the body's immune system's stress response following surgery, but laparoscopic surgery promotes the early restoration of immunological function due to less physical trauma. Laparoscopic surgery for colorectal cancer patients is less stressful and more useful than standard laparotomy, as shown by the much higher incidence rate of problems in the control group. In addition, there was no significant differences in postoperative survival rates and recurrence rates between the two groups, suggesting that concurrent laparoscopic surgery is safe and feasible for colorectal cancer patients.

However, the limitation of this study is that the sample size of the study is small, and the comparison of the two groups cannot exclude the bias of the results.

## 5. Conclusion

Laparoscopic surgery has fewer postoperative complications, shorter hospital stay, lower inflammatory factor expression, less stress response, better immune function, less trauma, and faster recovery, bringing patients a higher quality of life.

## Figures and Tables

**Figure 1:** Levels of inflammatory factors in serum before/after surgery in 2 groups. ^∗^*P* < 0.05, compared to preoperative levels; ^#^*P* < 0.05, compared to the control group.

**Figure 2:** Stress response before and after surgery in 2 groups. ^∗^*P* < 0.05, compared to preoperative levels; ^#^*P* < 0.05, compared to the control group.

**Figure 3:** Levels of immune indexes before and 10 d after the surgery in 2 groups. ^∗^*P* < 0.05, compared to preoperative levels; ^#^*P* < 0.05, compared to the control group.

**Figure 4:** Comparison of 2-year postoperative survival between the two groups.

**Table 1:** Comparison of the perioperative conditions between the two groups.

Group	Postoperative exhaust time (min)	Operation time (min)	Recovery time (d)	Hospital stay (d)	Intraoperative bleeding (mL)
Observation	68.6 ± 6.3	150.0 ± 21.4	1.8 ± 0.4	9.7 ± 2.4	79.4 ± 22.6
Control	70.1 ± 10.3	121.7 ± 25.2	2.7 ± 0.6	13.2 ± 4.1	151.35 ± 11.56
*t*	10.229	4.215	3.109	5.018	14.253
*P*	>0.05	<0.001	<0.005	<0.001	<0.001

RETRACTED

**Table 2:** Comparison of complication rates in the 2 groups.

Groups	*N*	Incision infection		Anastomotic leakage		Bleeding		Urinary infection		Total incidence rate	
		*N*	%	*N*	%	*N*	%	*N*	%	*N*	%
Control	48	3	6.25	2	4.17	2	4.17	2	4.17	9	18.75
Observation	47	1	2.13	0	0	1	2.13	0	0	2	4.26

## Data Availability

Dara analyzed in this study are available from the corresponding author upon reasonable request.
